# Segnet Network Algorithm-Based Ultrasound Images in the Diagnosis of Gallbladder Stones Complicated with Gallbladder Carcinoma and the Relationship between P16 Expression with Gallbladder Carcinoma

**DOI:** 10.1155/2021/2819986

**Published:** 2021-12-21

**Authors:** Liang Xue, Xiaohui Wang, Yong Yang, Guodong Zhao, Yanzhen Han, Zexian Fu, Guangxin Sun, Jie Yang

**Affiliations:** ^1^Department V of General Surgery, Affiliated Hospital of Hebei Engineering University, Handan 056002, Hebei, China; ^2^Endocrine Department, Affiliated Hospital of Hebei Engineering University, Handan 056002, Hebei, China

## Abstract

The study focused on how to improve the diagnostic coincidence rate of patients with gallbladder stones and gallbladder cancer based on an optimized Segnet network algorithm and the relationship of gallbladder cancer with multiple tumor suppressor 1 (P16). 300 patients diagnosed with gallbladder cancer in the hospital were selected as the research subjects. The pyramid pooling operation was incorporated into the original Segnet network algorithm, and its performance was evaluated, factoring into the intersection of union (IoU), algorithm precision (Pre), and recall rate (Recall). After 8 hours of fasting, conventional ultrasound and contrast-enhanced ultrasound examinations were performed, and the images were evaluated by three experienced ultrasound diagnosticians. The positive signal of P16 immunohistochemical staining was brownish yellow, which was generally concentrated in the nucleus, and a small part was located in the cytoplasm. In each slice, ten visual fields were selected. Then, they were observed under a high-power mirror, and the number was counted. It was found that the optimized Segnet network algorithm increased the IoU by 7.3%, the precision by 8.2%, and the recall rate by 11.1%. The diagnostic coincidence rates of conventional ultrasound and contrast-enhanced ultrasound examinations for gallbladder cancer were 78.13% (25/32) and 87.5% (25/32), respectively. The positive expression rate of P16 in gallbladder adenocarcinoma (47.06%) was significantly lower than that of acute cholecystitis with gallbladder stones (84.38%) and gallbladder polyps (67.16%) (*P* < 0.05). The positive expression rate of P16 in patients with stage III and stage IV (33.33% and 40%) was significantly lower than that in patients with stages I and II (87.5% and 80%) (*P* < 0.05). The positive expression rate of P16 in high differentiation (86.67%) was significantly higher than that of moderate differentiation (40%) and poor differentiation (28.57%) (*P* < 0.05). In short, contrast-enhanced ultrasound can effectively improve the diagnostic coincidence rate of gallbladder cancer, and the expression of P16 in gallbladder cancer is closely related to tumor staging and differentiation.

## 1. Introduction

Gallbladder carcinoma, mainly adenocarcinoma, is a common malignant tumor in the extrahepatic biliary system [1]. In China, the average age of the onset of gallbladder cancer is approximately 56 years. Generally speaking, gallbladder cancer is more common in women. In addition, more than 85% of clinical gallbladder cancer patients have gallbladder stones [2]. The incidence of gallbladder cancer in patients with gallbladder stones is about 7 times higher than that of people without gallbladder stones. Among patients with gallbladder stones, the risk of gallbladder cancer in patients with a single gallbladder stone greater than 3 cm in diameter is 10 times that of patients with a gallbladder stone less than 1 cm in diameter. Therefore, the cause of gallbladder cancer may be related to gallbladder stones [3]. The P16 gene, also known as multiple tumor suppressor 1 (MTS-1) gene, is a new type of tumor suppressor gene located on human chromosome 92P1. When the P16 protein is expressed at a low level, it will cause cell disorders and abnormal cell growth, and ultimately, it will lead to the formation of tumors [4].

For a long time, the main methods to diagnose gallbladder cancer included conventional ultrasound, computerized tomography (CT), endoscopic ultrasound, and magnetic resonance imaging (MRI) [5]. Conventional ultrasound can make accurate judgments on the morphological changes of gallbladder cancer, such as whether the size, location, and shape are regular, whether the bile duct is dilated, the degree of dilation, and the invasion of the adjacent tissue and lymph node metastasis, and it is recognized as the first choice to diagnose malignant tumors of the biliary system. Its diagnostic coincidence rate is approximately 80% [6]. Contrast-enhanced ultrasound can specifically diagnose tumors with rich and poor blood supply, and especially in the parenchymal stage, it can comprehensively scan the surrounding tissue of gallbladder cancer and detect lesions that conventional ultrasound cannot find [7]. Contrast-enhanced ultrasound uses a contrast agent to perfuse the tissue. The peak time (TTP), peak intensity (PI), contrast agent perfusion rate, and other related parameters are recorded to determine the benign and malignant tumors. It significantly improves the diagnostic coincidence rate [8].

Deep learning can extract the essential features of the target by network training on a large amount to elevate the classification accuracy. During the training, it can not only automatically learn but also automatically modify the learning parameters [9]. In this research, a Segnet algorithm was proposed that can reduce the running time of the model while keeping the detection accuracy unchanged. The Segnet algorithm can store the pooled index, avoid saving the feature map of the decoded part, and save memory [10].

The innovation of this study was to propose a new Segnet algorithm to process the conventional two-dimensional ultrasound image of 300 patients with gallbladder stones and gallbladder cancer. The immunohistochemical method was used to detect the expression level of the P16 protein in the cancer tissue. The primary objective of the study was to explore the accuracy, specificity, and sensitivity of contrast-enhanced ultrasound in the diagnosis of gallbladder cancer, as well as the relationship between the P16 protein expression and the tumor to fully understand the mechanism of gallbladder cancer and provide an evidence-based basis for the clinical diagnosis and treatment of gallbladder cancer.

## 2. Materials and Methods

### 2.1. Research Subjects

In the study, 300 patients diagnosed with gallbladder cancer in the hospital from October 15, 2017, to April 25, 2021, were selected as the research subjects, including 135 males and 165 females, with an average age of (56.82 ± 12.74) years. Inclusion criteria include those (I) aged over 50, (II) suffering from gallbladder stones for more than five years, (III) with the diameter of stones greater than 2 cm, (IV) with the local gallbladder wall thickened, and (V) with gallbladder polyps greater than 1 cm. The clinical symptoms included dull pain, abdominal distension, indigestion, nausea, and vomiting. The experiment has been approved by the ethics committee of the hospital. The patients and their families understood the research and signed an informed consent form.

### 2.2. Segnet Network Algorithm

The Segnet network algorithm mainly includes an encoding network and a decoding network. It can completely retain the feature information of the image, reduce the number of training parameters, shorten the training time, and display high-precision semantic segmentation images. The Segnet network algorithm comprises the convolutional layer, the normalization layer, the activation function, and the pooling layer (Figure 1).

The Segnet network algorithm structure has a symmetrical structure, with the left side of the network representing the encoding network and the right side representing the decoding network [11]. In the Segnet network, the pooling layer and the upsampling layer are used for image segmentation. The feature extraction of the target is completed by the left convolution layer, i.e., the encoding network. The pooling layer is used mainly to shrink the picture and perform deconvolution and upsampling operations [12]. Deconvolution is to make the classification features of the image more obvious. Upsampling is to restore the image to the same size as the input image. The encoding network extracts the features of the segmented image, transmits it to the decoding network, and outputs the semantic segmentation image (Figure 2).

In the training process, the linear expression cannot fully meet the actual needs, and the Relu function is often used for fitting. The Relu function is easy to calculate and fast to converge, and it is expressed as follows:

(1) $$\begin{array}{c} \text{f}\left(\text{x}\right)=\left\{\begin{array}{cc} x, & x>0,\\ 0, & x\leq 0. \end{array}\right. \end{array}$$

When the input signal ≤0, the output is 0. When the input signal *x* > 0, the output is equal to the input.

### 2.3. Pyramid Pooling Operation

In the original segnet network, the pooling operation will cause the loss of some high-frequency components in the image, produce a purification module, and lose the pixel position and spatial information (Figure 3). To avoid this problem, the pyramid pooling operation is introduced. The pyramid pooling module uses different coarse and fine scales to fuse features, and the output of different scales includes feature maps of various sizes. It avoids producing fuzzy blocks as much as possible and retains the original features extracted by the convolutional neural network (CNN) (Figure 4).

### 2.4. Evaluation Indicators of Experimental Results

There are three evaluation indicators to determine the accuracy of feature extraction. The first is the intersection of union (IoU). It represents the degree of overlap between the candidate area generated when detecting the target and the original marked area, and it is expressed as follows:

(2) $$\begin{array}{c} \text{IoU}=\frac{T1}{T1+S1+S2}, \end{array}$$

where T1 represents a correctly detected nontarget feature, S1 represents a nontarget feature that is erroneously detected as a target feature, and S2 represents a target feature that is erroneously detected as a nontarget feature.

The second is the precision (Pre), which is the percentage of real target pixels in the detected target features, and it is expressed as follows:

(3) $$\begin{array}{c} \text{Pre}=\frac{T1}{T1+S2}, \end{array}$$

where *T*1 represents a correctly detected nontarget feature, and S2 represents a target feature that is incorrectly detected as a nontarget feature.

The third is the recall rate (Recall). It is the ratio of the detected real target pixels to all the ultrasound samples of the test set and is expressed as follows:

(4) $$\begin{array}{c} \text{Recall}=\frac{T1}{T1+T2}, \end{array}$$

where *T*1 represents the nontarget feature that is correctly detected, and *T*2 represents the target feature that is correctly detected.

### 2.5. Ultrasonic Diagnostic Equipment

After 8 hours of fasting, patients with gallbladder cancer underwent a routine ultrasound examination. The patient was in a supine position to have the multisection examination of the upper abdomen, and the location, number, size, shape, boundary, and thickness of the gallbladder wall were recorded. Color ultrasound diagnostic apparatus was used for contrast-enhanced ultrasound, and an abdominal probe with a frequency of 3.5 MHz was used to detect the blood flow signal and shape of the lesion and determine the blood flow velocity. After angiography, three experienced ultrasound diagnosticians evaluated the images independently.

### 2.6. Immunohistochemical Staining Procedure and Result Judgment

The P16-positive gastric cancer tissue was used as a positive control, and the phosphate buffered saline (PBS) instead of P16 primary antibody was used as a negative control. The specific steps were as follows:

Firstly, after being dewaxed and hydrated, the paraffin sections were rinsed with PBS (PH = 7.4) three times for 3 minutes each time. Then, according to the requirements of each antibody, the tissue antigen was repaired accordingly. Each slice was immersed in 50uL peroxidase blocking solution to incubate for 10 minutes at room temperature to block the activity of endogenous peroxidase. Then, it was rinsed with PBS three times for 3 minutes each time. Next, each slice was immersed in 50uL normal nonimmune animal serum to incubate for 10 minutes at room temperature. Subsequently, the serum was removed, and each slice was immersed in 50uL of the primary antibody to incubate for 60 minutes at room temperature. Again, it was rinsed with PBS three times for 3 to 5 minutes each time. After the PBS solution was removed, each slice was immersed in 50uL biotin-labeled secondary antibody to incubate for 10 minutes at room temperature. Then, it was rinsed with PBS three times for 3 minutes each time. After the PBS solution was removed, each slice was immersed in 50uL streptavidin-peroxidase solution to incubate for 10 minutes at room temperature. Then, it was rinsed with PBS three times for 3 minutes each time. After the PBS solution was removed, each slice was immersed in 100uL of freshly prepared diaminobenzidine (DAB) solution and observed under a microscope for 3 to 10 minutes. Next, it was rinsed with tap water and stained with hematoxylin, followed by rinsing with PBS or tap water to return to blue. DAB was used for color development. The slices were dehydrated and dried with gradient alcohol, cleared with xylene, and mounted with neutral gum.

The positive signal of P16 immunohistochemical staining was brownish-yellow, generally concentrated in the nucleus, with a small part in the cytoplasm. In each slice, 10 fields of view were selected, which were then observed under a high-power mirror to count the number. More than 60% of the cells in the field of view with brown-yellow particles was defined as strong positive (+++), 30% to 60% of the cells with brown-yellow particles was defined as positive (++), 5% to 30% of cells with brown-yellow particles was defined as weakly positive (+), and no obvious brown particles in the cell were defined as negative (-). A weak positive expression or above was considered a positive expression.

### 2.7. Statistical Methods

In this study, SPSS21.0 statistical software was used for statistical analysis of the result data. The calculated data that conformed to the normal distribution were represented by the mean standard deviation ($\bar{x}$ ± *s*), and the calculated data that did not conform were represented by the percentage (%). The comparison of counting data adopts *χ*^2^ test. *P* < 0.05 indicated that the difference was significant.

## 3. Results

### 3.1. Performance of the Segnet Network Algorithm

The Segnet and the optimized Segnet with the pyramid model were trained separately.  Figure 5 shows the loss value/accuracy change curve of the training set and the validation set.  Figure 6 shows the semantic segmentation network. According to the result data, the optimized Segnet network algorithm of the pyramid pooling operation increased the IoU by 7.3%, the precise (Pre) by 8.2%, and the recall rate (Recall) by 11.1%. It suggested that the semantic segmentation model with pyramid pooling elevated the accuracy and speed of target extraction.

### 3.2. General Information of the Subjects

There were 300 patients with gallbladder cancer, including 135 males and 165 females, ranging in age from 50 to 75 years. Pathological examination showed 32 cases of gallbladder malignant tumors, of which gallbladder adenocarcinoma accounted for 53.12% (17 cases), gallbladder squamous cell carcinoma accounted for 25% (8 cases), gallbladder adenosquamous carcinoma accounted for 15.63% (5 cases), and gallbladder villous cystic glands tumor accounted for 6.25% (2 cases). There were 168 cases of benign gallbladder lesions, including 40% (67 cases) of gallbladder polyps, 11.31% (19 cases) of gallbladder adenoma, 8.33% (14 cases) of biliary sludge, 19.04% (32 cases) of acute cholecystitis with gallbladder stones, and 21.43% (36 cases) of chronic cholecystitis with gallbladder stones (Figure 7).

### 3.3. Results of Conventional Ultrasound Examination

25 cases of gallbladder cancer were detected by conventional ultrasound examination. The diagnosis coincidence rate was 78.13% (25/32). 4 cases of nodular gallbladder carcinoma had nodular protrusions in the gallbladder cavity, wide basement, irregular edges, and heterogeneous internal echoes. The abnormal central echoes caused by stones, air, or necrosis were noted (Table 1). In 5 cases of thick-walled gallbladder carcinoma, the gallbladder wall was locally thickened or diffusely unevenly thickened, showing hyperechoic (more common) or hypoechoic signals, and the entire gallbladder was stiff, deformed, and the wall was rough or irregular. In 5 cases of solid gallbladder carcinoma, the entire gallbladder showed disordered low-echo or medium-echo solid masses, and the dark areas in the gallbladder cavity disappeared, often accompanied by gallbladder stones. There were 6 cases of mixed gallbladder carcinoma, and both thick-walled and nodular types were noted (Figure 8).

### 3.4. Results of Contrast-Enhanced Ultrasound Examination

28 cases of gallbladder cancer were examined by contrast-enhanced ultrasound, and the diagnosis coincidence rate was 87.5% (25/32). For patients with gallbladder stones combined with gallbladder cancer, the mass was large, the boundary was not clear, and the surrounding halo was visible. There were irregular liquid dark areas inside, the mass was adjacent to the gallbladder, and the boundary with the gallbladder was not clear (Figure 9; Table 2).

### 3.5. Immunohistochemical Staining Results of P16

The positive expression of P16 was mainly concentrated in the nucleus and cytoplasm, with brownish-yellow particles, and some cell membranes were also stained (Figure 10).

### 3.6. Expression of P16 in Lesions of Gallbladder Carcinoma

In 17 cases of gallbladder adenocarcinoma, the positive expression rate of P16 was 47.06%. In 67 cases of gallbladder polyps, the positive expression rate of P16 was 67.16%. In 32 cases of acute cholecystitis with gallbladder stones, the positive expression rate of P16 was 84.38%. In 36 cases of chronic cholecystitis with gallbladder stones, the positive expression rate of P16 was 81.56%. The positive expression rate of P16 in gallbladder adenocarcinoma was significantly lower than that in patients with other gallbladder lesions, and the difference was significant (*P* < 0.05) (Figure 11).

### 3.7. The Relationship between the Positive Expression of P16 and Pathological Features

As per the clinical staging of gallbladder cancer, there are 8 cases in stage I, 5 cases in stage II, 9 cases in stage III, and 10 cases in stage IV. The positive expression rate of P16 in the patients of stages III and IV (33.33% and 40%) was significantly lower than that of the patients of stages I and II (87.5% and 80%), and the difference is significant (*P* < 0.05) (Figure 12).

According to the results of tumor differentiation, 7 cases were poorly differentiated, 10 cases were moderately differentiated, and 15 cases were highly differentiated. The positive expression rate of P16 in the high differentiation (86.67%) was significantly higher than that of moderate differentiation (40%) and poor differentiation (28.57%), and the difference was significant (*P* < 0.05) (Figure 13).

## 4. Discussion

Gallbladder cancer is a common malignant tumor of the biliary system, and its incidence has been increasing in recent years. Gallbladder cancer combined with gallbladder stones continuously stimulates the gallbladder wall mucosa, causing the abnormal proliferation of mucosal epithelial cells and cholestasis. Gallbladder cancer lacks specific clinical manifestations in the early stage and has similar symptoms of gallbladder stones. Therefore, when it is discovered, it is already in the middle and late stages when the best treatment opportunity has been lost [13,14]. At present, the early diagnosis of gallbladder cancer combined with gallbladder stones is a clinical problem that needs to be solved urgently.

Conventional ultrasound examination is easy to operate, noninvasive, low in price, and easy to be accepted by patients. It is recognized as the first choice for the diagnosis of gallbladder cancer [15]. However, because of the limitations of the technology itself, the microvessels of the lesion cannot be well-evaluated. In this study, 25 cases of gallbladder cancer were detected by conventional ultrasound, and the diagnosis coincidence rate was 78.13% (25/32), which was consistent with the research results of Rana et al. (2016) [16]. There were a total of 7 cases of missed and misdiagnosed cases. The main reasons were as follows: firstly, there is a certain amount of bile mud and viscous bile deposited in the gallbladder, and they do not move when the body position changes. Secondly, the thickness of the normal gallbladder wall is approximately 2 mm. When it is greater than 4 mm, the stone has an arc shape, and it is easy to misdiagnose the gallbladder with a thickened gallbladder wall and gallbladder cancer as chronic cholecystitis and gallstone disease. Thirdly, there are many organs around the gallbladder and abundant vessels. After gallbladder cancer has infiltrated, the outline of the gallbladder is unclear, and it is easy to be misdiagnosed as a tumor in the surrounding tissue.

Contrast-enhanced ultrasound technology is an imaging technology to understand the anatomy of tumor blood vessels. It can enhance the backscattered echo of the cells and improve the diagnostic coincidence rate. However, the low-resolution results in the unclear intima of large blood vessels, and it is unable to identify tiny blood vessels [17]. In this study, 28 cases of gallbladder cancer were detected by contrast-enhanced ultrasound, and the diagnosis coincidence rate was 87.5% (25/32). Contrast-enhanced ultrasound can observe the blood flow characteristics of the lesions of gallbladder cancer patients in real time, accurately display the spatial distribution of vascular perfusion, and significantly improve the signal ratio of detection. In this study, it can accurately detect the invasive growth of gallbladder tumors, providing a theoretical basis for the diagnosis of gallbladder cancer.

The P16 gene is a tumor suppressor gene directly involved in the negative feedback regulation of the cell cycle, and its level is closely related to the cell cycle [18,19]. When the P16 gene has mutations or deletions, it will lead to a low expression or the inactivation of the P16 protein, leading to cell cycle disorders [20]. In this study, the positive expression rate of P16 in gallbladder adenocarcinoma (47.06%) was significantly lower than that of acute cholecystitis with gallbladder stones (84.38%) and gallbladder polyps (67.16%) (*P* < 0.05). It showed that P16 was obviously missing in gallbladder cancer tissue, and the deletion and mutation of the P16 gene would lead to the occurrence of gallbladder cancer. The positive expression rate of P16 in the high differentiation (86.67%) was significantly higher than that in the middle differentiation (40%) and poor differentiation (28.57%) (*P* < 0.05), indicating that the positive expression of P16 protein in the gallbladder cancer tissue was related to the degree of tissue differentiation.

## 5. Conclusion

In this study, the ultrasound images based on the optimized Segnet network algorithm were used to diagnose 300 patients with gallbladder stones and gallbladder cancer. It was found that contrast-enhanced ultrasound can effectively improve the diagnostic coincidence rate of gallbladder cancer, and the expression of P16 in gallbladder cancer was closely related to tumor staging and differentiation. However, some limitations in the study should be noted. The sample size is small, which will reduce the power of the study. In the follow-up, an expanded sample size is necessary to strengthen the findings of the study. In conclusion, ultrasound imaging as a new imaging technology has guiding significance in the early diagnosis and identification of gallbladder cancer.

## Figures and Tables

**Figure 1:** Structure of the Segnet network algorithm.

**Figure 2:** Relu function.

**Figure 3:** Original pooling operation.

**Figure 4:** Pyramid pooling module.

**Figure 5:** Loss value/accuracy curve of training set and validation set. (a) Segnet network algorithm. (b) Optimized Segnet network algorithm.

**Figure 6:** Comparison of semantic segmentation networks.

**Figure 7:** The pathological examination results. (a) Malignant tumor of the gallbladder. (b) Benign lesions of the gallbladder.

**Figure 8:** Conventional ultrasound examination results. (a) Nodular type, with moderate and weak echoes. (b) Thick-walled type, with diffuse and uneven thickening of the gallbladder wall. (c) Solid type, with an enlarged gallbladder, strong echo group with sound shadow. (d) Mixed type, the gallbladder wall was thickened regularly with papillary protrusions.

**Figure 9:** Contrast-enhanced ultrasound examination. (a) The patient was a 62-year-old male with a history of gallbladder stones for 5 years and epigastric pain for 5 days. Contrast-enhanced ultrasound examination of the abdomen showed that the continuity of the gallbladder wall was locally interrupted, and a slightly strong echogenic nodule protruding into the cavity was seen near the bottom. (b) The patient was a 55-year-old female with dull pain in the upper abdomen for half a year. Contrast-enhanced ultrasound examination of the abdomen showed the thickening of the gallbladder wall, and a moderate echogenic mass filled the cyst cavity at the bottom of the gallbladder. (c) The patient was a 53-year-old female with abdominal pain for 3 days. Contrast-enhanced ultrasound examination of the abdomen showed that the gallbladder volume increased significantly, and a solid mass with irregular shape was seen in the cyst cavity. (d) The patient was a 64-year-old female with a history of gallbladder stones for 5 years and epigastric pain for 5 days. Contrast-enhanced ultrasound examination of the abdomen showed clear boundaries of gallbladder lesions and irregular thickening of the cyst wall.

**Figure 10:** Results of immunohistochemical staining. (a) P16 was negatively expressed (×200). (b) P16 was weakly expressed (×200). (c) P16 was positively expressed (×200). (d) P16 was strongly positively expressed (×200).

**Figure 11:** Positive expression of P16 in the lesions of gallbladder cancer. ^*∗*^indicates that compared with gallbladder adenocarcinoma, the difference was significant, i.e., *P* < 0.05.

**Figure 12:** The relationship between the positive expression of P16 and tumor stage. ^*∗*^means that compared with stage (I), the difference was significant, i.e., *P* < 0.05.

**Figure 13:** The relationship between the positive expression of P16 and the degree of differentiation. ^*∗*^indicates that compared with high differentiation, the difference was significant, i.e., *P* < 0.05.

**Table 1:** Conventional ultrasound examination results.

	Gallbladder malignant tumor	Benign gallbladder disease
Pathological diagnosis (case)	32	168
Conventional ultrasound diagnosis (case)	25	161
Diagnosis coincidence rate (%)	78.13	95.83

**Table 2:** Results of contrast-enhanced ultrasound examination.

	Gallbladder malignant tumor	Benign gallbladder disease
Pathological diagnosis (case)	32	168
Contrast ultrasound diagnosis (case)	28	166
Diagnosis coincidence rate (%)	87.5	98.8

## Data Availability

The data used to support the findings of this study are available from the corresponding author upon request.
